# Racial Disparity Amongst Stroke Patients During the Coronavirus Disease 2019 Pandemic

This article has been retracted.

**DOI:** 10.7759/cureus.10369

**Published:** 2020-09-10

**Authors:** Hammad Ghanchi, Tye Patchana, James Wiginton, Jonathan D Browne, Ai Ohno, Ronit Farahmandian, Jason Duong, Vladimir Cortez, Dan E Miulli

**Affiliations:** 1 Neurosurgery, Riverside University Health System Medical Center, Moreno Valley, USA; 2 Neurosurgery, California University of Science and Medicine, San Bernardino, USA; 3 Neurosurgery, Riverside University Health System Medical Center, Rancho Cucamonga, USA; 4 Neurosurgery, Arrowhead Regional Medical Center, Colton, USA

**Keywords:** covid, covid 19, stroke, racial disparity

## Abstract

Introduction

The global coronavirus disease 2019 (COVID-19) pandemic has had deleterious effects on our healthcare system. Lockdown measures have decreased the number of patients presenting to the hospital for non-respiratory illnesses, such as strokes. Moreover, there appears to be a racial disparity among those afflicted with the virus. We sought to assess whether this disparity also existed for patients presenting with strokes.

Methods

The Get with the Guidelines National Stroke Database was reviewed to assess patients presenting with a final diagnosis of ischemic stroke, transient ischemic attack (TIA), subarachnoid hemorrhage (SAH), or spontaneous/nontraumatic intraparenchymal hemorrhage (IPH). The period of February - May 2020 was chosen given the surge of patients affected with the virus and national shutdowns. Data from this same time during 2019 was used as the control population. Our hospital numbers and four additional regions were assessed (California hospitals, Pacific State hospitals, Western Region hospitals, and all hospitals in the United States). Patients were categorized by race (White, Black/African American, Asian, Native American, Hispanic) in each cohort. The primary endpoint of this study is to compare whether there was a significant difference in the proportion of patients in each reported racial category presenting with stroke during the COVID-19 pandemic caused by severe acute respiratory syndrome coronavirus 2 (SARS-CoV-2).

Results

A downward trend in total number of patients was noted in all five regional cohorts assessed. A statistically significant increase in the number of Black and Hispanic patients presenting with strokes was noted in California, Pacific hospitals, Western hospitals, and all hospitals in the United States during various months studied comparing 2020 to 2019. A statistically significant increase in the Hispanic population was noted in February and March in all California hospitals (p=0.005 and 0.02, respectively) and Pacific Coast hospitals (p=0.005 and 0.039, respectively). The Western region and all national hospitals noted a significant increase in strokes in the Hispanic population in April (p=0.039 and 0.023, respectively). A statistically significant increase of strokes in the Black population was noted in April in Pacific hospitals, Western region hospitals, and all national hospitals (p=0.039, 0.03, and 0.03, respectively).

Conclusion

The COVID-19 pandemic has adversely affected certain racial groups more than others. A similar increase is noted in patients presenting with strokes in these specific racial populations. Moreover, lack of testing for the SARS-CoV-2 virus may be missing a possible link between racial disparity for patients infected with the virus and patients presenting with stroke. The authors advocate for widespread testing for all patients to further assess this correlation.

## Introduction

The coronavirus disease 2019 (COVID-19) pandemic, caused by the severe acute respiratory syndrome coronavirus 2 (SARS-CoV-2), has affected many aspects of healthcare, including stroke care. Significant racial disparities among populations affected by COVID-19 have recently made headlines. Some sources have also cited SARS-CoV-2 as a possible cause of stroke [1]. Nationally, Hispanics and Blacks are disproportionately represented among laboratory-confirmed COVID-19 cases [2]. As of June 27, age-adjusted COVID-19-associated hospitalization rates were highest among people who are non-Hispanic American Indian/Alaska Native, non-Hispanic Black, and Hispanic/Latino according to the COVID-19-Associated Hospitalization Surveillance Network (COVID-NET) [3]. Higher rates of COVID-19 deaths were reported in counties with a high Black population, especially in rural and small metro counties [4]. 

This is not the first time in history that racial disparity has existed in medicine; surgeries on Black women without anesthesia by Dr. Sims [5] and the Tuskegee syphilis study are two examples of racism and prejudice that have caused distrust towards the medical sciences among this population [6]. There are no known unethical practices during the recent pandemic, however, this lingering mistrust can lead to delayed presentation in the setting of stroke and render Black patients to be ineligible for receiving intravenous tissue plasminogen activator (IV-tPA) treatment [7]. Despite the national decline in the mortality rate from stroke, it remains the second leading cause of death in Blacks [8]. Moreover, Black individuals have been shown to have a higher mortality rate [9] and a higher chance of experiencing disability [10] following a stroke compared to Whites. Furthermore, the American Heart Association (AHA) Stroke Council Scientific Oversight Committee has reported a history of racial discrepancies in stroke risk factors, incidence, prevalence, and symptom recognition [11].

Given the recent pandemic and racial disparity among patients afflicted with SARS-CoV-2 and the possible link of this virus and cerebrovascular accidents (CVA), we sought to analyze whether there was a disparity for stroke patients presenting to hospitals during this time using the Get with the Guidelines (GWTG) National Stroke Database. The primary endpoint of this study is to assess whether disparity exists at our own hospital. We also wanted to expand this scope to the regional and national levels to assess for any possible racial disparities.

## Materials and methods

The GWTG stroke registry at our institution, a Level 1 primary stroke center certified by the Healthcare Facilities Accreditation Program, was retrospectively reviewed to assess the impact of the SARS-CoV-2 outbreak on the number of patients presenting with stroke to our hospital. Demographics with regards to patients' race were collected. Data were stratified by date and comparison was made between the COVID-19 period (February - May 2020) and similar timeframe pre-COVID-19 (February - May 2019). The months preceding the COVID-19 period (October 2019 - Janurary 2020) were avoided as a control as it is hard to know whether SARS-CoV-2 was propagating in the population during this time. The GWTG database was used to review records at our hospital, all California hospitals, West and Pacific regions, and all hospitals nationally.

Patients presenting to these hospitals with a final diagnosis of ischemic stroke, transient ischemic attack (TIA), subarachnoid hemorrhage (SAH), or spontaneous/nontraumatic intraparenchymal hemorrhage (IPH) were reviewed. After data was extracted from the database, the cohorts were stratified into five groups: (a) our hospital, (b) all California hospitals, (c) all Pacific Coast hospitals (Alaska, Washington, Oregon, California, and Hawaii), (d) all Western hospitals (Pacific plus Montana, Idaho, Wyoming, Nevada, Utah, Colorado, Arizona, and New Mexico), and (e) all hospitals in the United States that submit data to the registry. Among these groups, the number and relative proportion of each reported race (White, Black/African American, Asian, Native American, or Hispanic) were reviewed each month during COVID-19 and a similar time frame pre-COVID-19. Proportions were chosen instead of volume of patients to limit any confounding decreases/changes in the number of patients in each time frame as recent data has suggested a decrease in total number of stroke patients presenting to the hospital during this time [12].

The primary endpoint of this study is to compare whether there was a significant difference in the proportion of patients in each reported racial category presenting to our institution with stroke during the COVID-19 pandemic caused by SARS-CoV-2. The same analysis was conducted for the Pacific hospitals, Western hospitals, and all national hospitals. Statistical analysis was performed using Z-Test to compare the proportions for all races for any significant difference month by month (i.e. February 2019 compared to February 2020, March 2019 compared to March 2020, etc.).

## Results

There was an average of 51.75 patients per month in 2019 and 49 patients per month in 2020 during the time frame studied at our hospital. This downward trend in 2020 compared to 2019 in total patients per month was echoed in all the groups studied (California, Pacific, Western Region, and National). The total number of patients in each subgroup can be viewed in the Appendix. To remove the confounding effect of decreased patient numbers, as this decrease became more evident on the regional and national levels (i.e. mean of 57,864.5 patients nationally February through May 2019 versus 45,927.75 patients during the same months in 2020) during the COVID-19 months, the percentage of each race presenting to each hospital category was calculated (see Appendix). 

Looking at our hospital’s local population, a significant difference in Native Hawaiian/Pacific Islander population was noted in February 2020 compared to 2019 (p=0.01) but other racial cohorts remained similar (Table 1). Data for Asian and American Indian or American Native populations were insufficiently powered to perform statistical analysis. Expanding the scope to include all California hospitals, a significant difference was noted again in the Native Hawaiian/Pacific Islander population in February 2020 compared to the prior year (p<0.01). The Hispanic population also showed a significant difference for the months of February and March (p=0.005 and p=0.02, respectively). The remainder of racial cohorts in California remained stable during the studied time studied.

**Table 1:** P-Values Comparing Racial Proportions Monthly 2019 to 2020 Abbreviations: AA: African American, AI or AN: American Indian or American Native, NH or PI: Native Hawaiian or Pacific Islander, Feb: February, Mar: March, Apr: April

		White	Black or AA	Asian	AI or AN	NH or PI	Hispanic
Our Hospital							
	Feb	0.750	0.225	N/A	N/A	0.013	0.538
	Mar	0.250	0.775	N/A	N/A	0.988	0.463
	Apr	0.231	0.876	0.054	0.817	N/A	0.161
	May	0.552	0.431	N/A	N/A	0.175	0.345
All California							
	Feb	0.987	0.964	0.354	0.932	0.001	0.005
	Mar	0.265	0.450	0.516	0.640	0.537	0.020
	Apr	0.754	0.087	0.936	0.479	0.642	0.122
	May	0.546	0.901	0.113	0.631	0.656	0.311
Pacific Coast							
	Feb	0.944	0.947	0.266	0.996	0.634	0.005
	Mar	0.619	0.559	0.581	0.101	0.350	0.039
	Apr	0.765	0.039	0.917	0.568	0.856	0.073
	May	0.358	0.870	0.312	0.588	0.535	0.186
Western Region							
	Feb	0.992	0.850	0.307	0.994	0.621	0.185
	Mar	0.896	0.311	0.431	0.379	0.170	0.175
	Apr	0.920	0.030	0.809	0.359	0.743	0.039
	May	0.498	0.805	0.245	0.821	0.470	0.347
National							
	Feb	0.789	0.858	0.293	0.919	0.530	0.473
	Mar	0.946	0.030	0.678	0.918	0.301	0.649
	Apr	0.999	0.065	0.637	0.112	0.952	0.023
	May	0.873	0.263	0.082	0.929	0.237	0.652

When similar analysis was conducted for the Pacific Coast hospitals (Alaska, Washington, Oregon, California, and Hawaii), a significant difference was noted in the Black/African American cohort (p=0.039). The trend of significantly more Hispanic patients also existed in this cohort during February and March (p=0.005 and p=0.039, respectively). Differences in racial cohorts for all Western states (Pacific states plus Montana, Idaho, Wyoming, Nevada, Utah, Colorado, Arizona, and New Mexico) were only demonstrated during the month of April for Black/African Americans (p=0.03) and the Hispanic population (p=0.039). Finally, the national data for the United States demonstrated a statistically significant increase in the Black/African American population in March (p=0.03) and in April for the Hispanic population (p=0.023).

## Discussion

Racial disparities are well documented in all aspects of stroke as it relates to differences in stroke risk factors, incidence, prevalence, and symptom recognition in comparison to the White population [11]. While disparity in stroke may partially be explained by geography [13], neighborhood socioeconomic status [14], or age [15], there is substantial evidence emphasizing racial predisposition to stroke. The first-stroke risk at age 45 is 2.7 times higher in Black individuals compared to White individuals, with Black patients having higher rates of ischemic and hemorrhagic stroke [16]. In one cohort study, Black patients also had a 60% greater risk of recurrent stroke within two years compared to White patients, as well as higher prevalence of key vascular risk factors, including hypertension, diabetes mellitus, smoking, and high BMI [17]. Prevalence of underlying comorbidities and differences in leisure-time physical activity and diet may be contributing to the racial disparity among patients presenting with stroke prior to and during the COVID-19 period. Among patients hospitalized for COVID-19 with data on underlying conditions, 89.3% had at least one underlying condition according to the U.S. Centers for Disease Control and Prevention [18]. These included preventable vascular risk factors related to poor diet and physical inactivity, such as hypertension, cardiovascular disease, obesity, and diabetes [19]. Relative to non-Hispanic Whites, Blacks have historically been found to be less physically active [20] and have poorer diets [21]. This trend is consistent with the disproportionate increase in Blacks presenting with stroke on a national level in March 2020 from the prior year. In contrast, Hispanics have been found to have healthier diets than Whites [21-23] although poorer diets have been reported among those with high acculturation status [23]. This interaction between acculturation status and dietary behavior may be contributing to the difference in trend seen among Hispanic patients presenting with stroke at a regional versus national level.

As of late June 2020, age-adjusted COVID-19-associated hospitalization rates were highest among people who are non-Hispanic American Indian/Alaska Native, non-Hispanic Black, and Hispanic/Latino according to the COVID-19-Associated Hospitalization Surveillance Network (COVID-NET) [3]. Our study demonstrates a similar trend for patients presenting with stroke with the relative proportion of White patients decreasing on a national level in March 2020 with an increase in Black population to 17.04% compared to 16.59% from the prior year (p=0.03) and in April 2020 the Hispanic population increasing to 8.13% from 7.76% the prior year (p=0.023). A similar trend was also seen in California and the Pacific Coast hospitals with an increase in the Hispanic population in February and March 2020 compared to the prior year. In California, there was an increase from 18.82% to 20.72% (p=0.005) and 19.73% to 20.8% (p=0.02) in February and March, respectively. In the Pacific Coast hospitals, there was an increase from 14.81% to 16.31% (p=0.005) and 15.72% to 16.31% (p=0.039) in February and March, respectively. While not statistically significant, a similar upward trend was also seen in our institution in February 2020 compared to the prior year. This increase in number of strokes in February may be COVID-19-related as the virus was propagating prior to when precautions were placed in March at many institutions.

It has previously been reported that COVID-19 patients may present with ischemic stroke [24]. Influenza-like illnesses have also been linked to stroke [25]. While yet to be proven, there are several proposals on how COVID-19 may increase the risk of stroke. Angiotensin converting enzyme (ACE) II receptor is a functional receptor and entry point for SARS-CoV and SARS-CoV-2. Involved in cardiovascular homeostasis, the receptor is expressed on several vital tissues, including vascular endothelium, arterial smooth muscle, and the brain [26]. SARS-CoV infection appears to downregulate ACE II [27], which may contribute to increased stroke risk. Cardiac embolism from virus-related cardiac injury [28], hypercoagulability exhibited by elevated D-dimer levels [29], and inflammatory reactions due to cytokine storm [30] are other mechanisms in which COVID-19 may lead to increased risk of stroke. Stress from lockdown-induced isolation increases sympathetic release cytokines which affects the comorbidities of this end-organ disease. These factors amplify the effects of stroke in this population.

Furthermore, during the month of February 2020, the data demonstrate an increase in the total number of patients presenting with strokes in all subgroups (Appendix Table 2). Given the possibility of SARS-CoV-2 causing vascular injury, this rise may be attributed to early stages of the COVID-19 pandemic, i.e. SARS-CoV-2 was propagating in February in the United States possibly causing increase in stroke numbers. This rise in total numbers was then mitigated during the following months by the nationwide lockdowns and patient fears of contracting the infection. Testing for SARS-CoV-2 was not being performed at this time, so this postulation is difficult to prove. Moreover, given the possibility of carriers of this virus being asymptomatic from a respiratory standpoint, patients presenting with stroke may fall into this category.

Limitations

One major limitation of this study is the lack of widespread testing for SARS-CoV-2. The cause for the increase in the number of strokes in February 2020 before lockdown measures is uncertain but given the virus was circulating during this time along with the vascular injury it causes make it a possible suspect. Moreover, lack of widespread testing the months following also limits our ability to assess whether the increase in certain races being more adversely affected from the virus and increase in the number of strokes in the same ethic groups is related. Thus, we hope to advocate for universal testing for SARS-CoV-2 for all patients presenting to the hospital to further isolate possible carriers who are asymptomatic from a respiratory standpoint. Moreover, given the retrospective nature of this study, we are unable to retroactively implement these goals.

## Conclusions

The global COVID-19 pandemic has had many devastating effects on not only our economy and lifestyles, but also our healthcare system. Certain races are being more adversely affected than others from this virus due to the effects on the human physiology and the ability of the virus amplify the negative health effects of the comorbid conditions of stroke. The potential for this virus to cause strokes may be causing our observed increase in minority cerebrovascular accidents. Increase in stroke numbers prior to lockdowns may be related to early propagation of the virus. Further work is needed to assess this relationship as well as more widespread testing for SARS-CoV-2 to determine the true pathophysiology of this illness.

## Appendices

**Table 2:** Number of Patients in each subgroup Abbreviations: AA: African American, AI or AN: American Indian or American Native, NH or PI: Native Hawaiian or Pacific Islander, Feb: February, Mar: March, Apr: April

	White	Black or AA	Asian	AI or AN	NH or PI	Hispanic		
							Total	Mean
Our Hospital								
Feb 2019	28	8	0	0	0	19	55	51.75
Mar 2019	27	5	1	0	0	21	54	
Apr 2019	24	4	0	1	0	16	45	
May 2019	25	9	1	0	0	18	53	
Feb 2020	32	10	0	0	1	24	67	49
Mar 2020	23	6	0	1	0	19	49	
Apr 2020	21	1	2	0	0	16	40	
May 2020	21	3	0	0	0	16	40	
California								
Feb 2019	3667	548	617	28	26	1133	6019	6281.5
Mar 2019	3908	544	725	17	41	1287	6522	
Apr 2019	3801	521	675	20	33	1229	6279	
May 2019	3785	560	672	17	33	1239	6306	
Feb 2020	3742	519	662	19	58	1307	6307	5202.5
Mar 2020	3438	478	631	13	35	1207	5802	
Apr 2020	2773	418	456	15	22	947	4631	
May 2020	2485	337	398	16	24	810	4070	
Pacific States								
Feb 2019	5283	625	829	56	135	1204	8132	8555.25
Mar 2019	5707	638	986	38	123	1397	8889	
Apr 2019	5529	586	936	44	118	1303	8516	
May 2019	5579	650	952	44	128	1331	8684	
Feb 2020	5412	596	889	33	135	1377	8442	6989.5
Mar 2020	4971	553	854	44	113	1299	7834	
Apr 2020	4020	477	642	31	74	1010	6254	
May 2020	3537	387	544	33	73	854	5428	
Western States								
Feb 2019	7416	755	889	107	144	1501	10812	11413.75
Mar 2019	8066	791	1060	85	129	1706	11837	
Apr 2019	7793	761	1001	93	129	1583	11360	
May 2019	7936	808	1026	100	139	1637	11646	
Feb 2020	7686	759	962	78	147	1636	11268	9310
Mar 2020	6977	709	934	78	127	1538	10363	
Apr 2020	5548	606	693	71	85	1215	8218	
May 2020	5076	507	597	61	81	1069	7391	
National								
Feb 2019	38669	8921	1635	251	187	4231	53894	57864.5
Mar 2019	42430	9839	1902	258	182	4684	59295	
Apr 2019	41521	9610	1837	256	210	4497	57931	
May 2019	43101	10061	1898	297	186	4795	60338	
Feb 2020	40302	9191	1741	231	194	4429	56088	45927.75
Mar 2020	37265	8913	1655	200	170	4106	52309	
Apr 2020	28118	6737	1244	197	119	3224	39639	
May 2020	25545	6071	1135	162	119	2643	35675	

**Table 3:** Porportion of Patients in each Subgroup Abbreviations: AA: African American, AI or AN: American Indian or American Native, NH or PI: Native Hawaiian or Pacific Islander, Feb: February, Mar: March, Apr: April

	White	Black or AA	Asian	AI or AN	NH or PI	Hispanic	
							Total
Our Hospital							
Feb 2019	50.91%	14.55%	0.00%	0.00%	0.00%	34.55%	100%
Mar 2019	50.00%	9.26%	1.85%	0.00%	0.00%	38.89%	100%
Apr 2019	53.33%	8.89%	0.00%	2.22%	0.00%	35.56%	100%
May 2019	47.17%	16.98%	1.89%	0.00%	0.00%	33.96%	100%
Feb 2020	47.76%	14.93%	0.00%	0.00%	1.49%	35.82%	100%
Mar 2020	46.94%	12.24%	0.00%	2.04%	0.00%	38.78%	100%
Apr 2020	52.50%	2.50%	5.00%	0.00%	0.00%	40.00%	100%
May 2020	52.50%	7.50%	0.00%	0.00%	0.00%	40.00%	100%
California							
Feb 2019	60.92%	9.10%	10.25%	0.47%	0.43%	18.82%	100%
Mar 2019	59.92%	8.34%	11.12%	0.26%	0.63%	19.73%	100%
Apr 2019	60.54%	8.30%	10.75%	0.32%	0.53%	19.57%	100%
May 2019	60.02%	8.88%	10.66%	0.27%	0.52%	19.65%	100%
Feb 2020	59.33%	8.23%	10.50%	0.30%	0.92%	20.72%	100%
Mar 2020	59.26%	8.24%	10.88%	0.22%	0.60%	20.80%	100%
Apr 2020	59.88%	9.03%	9.85%	0.32%	0.48%	20.45%	100%
May 2020	61.06%	8.28%	9.78%	0.39%	0.59%	19.90%	100%
Pacific States							
Feb 2019	64.97%	7.69%	10.19%	0.69%	1.66%	14.81%	100%
Mar 2019	64.20%	7.18%	11.09%	0.43%	1.38%	15.72%	100%
Apr 2019	64.92%	6.88%	10.99%	0.52%	1.39%	15.30%	100%
May 2019	64.24%	7.49%	10.96%	0.51%	1.47%	15.33%	100%
Feb 2020	64.11%	7.06%	10.53%	0.39%	1.60%	16.31%	100%
Mar 2020	63.45%	7.06%	10.90%	0.56%	1.44%	16.58%	100%
Apr 2020	64.28%	7.63%	10.27%	0.50%	1.18%	16.15%	100%
May 2020	65.16%	7.13%	10.02%	0.61%	1.34%	15.73%	100%
Western States							
Feb 2019	68.59%	6.98%	8.22%	0.99%	1.33%	13.88%	100%
Mar 2019	68.14%	6.68%	8.95%	0.72%	1.09%	14.41%	100%
Apr 2019	68.60%	6.70%	8.81%	0.82%	1.14%	13.93%	100%
May 2019	68.14%	6.94%	8.81%	0.86%	1.19%	14.06%	100%
Feb 2020	68.21%	6.74%	8.54%	0.69%	1.30%	14.52%	100%
Mar 2020	67.33%	6.84%	9.01%	0.75%	1.23%	14.84%	100%
Apr 2020	67.51%	7.37%	8.43%	0.86%	1.03%	14.78%	100%
May 2020	68.68%	6.86%	8.08%	0.83%	1.10%	14.46%	100%
National							
Feb 2019	71.75%	16.55%	3.03%	0.47%	0.35%	7.85%	100%
Mar 2019	71.56%	16.59%	3.21%	0.44%	0.31%	7.90%	100%
Apr 2019	71.67%	16.59%	3.17%	0.44%	0.36%	7.76%	100%
May 2019	71.43%	16.67%	3.15%	0.49%	0.31%	7.95%	100%
Feb 2020	71.85%	16.39%	3.10%	0.41%	0.35%	7.90%	100%
Mar 2020	71.24%	17.04%	3.16%	0.38%	0.32%	7.85%	100%
Apr 2020	70.94%	17.00%	3.14%	0.50%	0.30%	8.13%	100%
May 2020	71.60%	17.02%	3.18%	0.45%	0.33%	7.41%	100%

## References

[1] Kalyanaraman Marcello R, Dolle J, Grami S (2020). Characteristics and outcomes of COVID-19 patients in New York City’s public hospital system. medRxiv.

[2] Stokes EK, Zambrano LD, Anderson KN (2020). Coronavirus Disease 2019 case surveillance - United States, January 22-May 30. MMWR Morb Mortal Wkly Rep.

[3] (2020). Data Visualization. https://www.cdc.gov/coronavirus/2019-ncov/covid-data/data-visualization.htm.

[4] Millett GA, Jones AT, Benkeser D (2020). Assessing differential impacts of COVID-19 on black communities. Ann Epidemiol.

[5] Ojanuga D (1993). The medical ethics of the “father of gynaecology”, Dr J Marion Sims. J Med Ethics.

[6] Dovidio JF, Penner LA, Albrecht TL, Norton WE, Gaertner SL, Shelton JN (2008). Disparities and distrust: the implications of psychological processes for understanding racial disparities in health and health care. Soc Sci Med.

[7] Hsia AW, Edwards DF, Morgenstern LB (2011). Racial disparities in tissue plasminogen activator treatment rate for stroke: a population-based study. Stroke.

[8] Towfighi A, Saver JL (2011). Stroke declines from third to fourth leading cause of death in the United States: historical perspective and challenges ahead. Stroke.

[9] Howard G, Howard VJ (2001). REasons for Geographic And Racial Differences in Stroke (REGARDS) Investigators. Ethnic disparities in stroke: the scope of the problem. Ethn Dis.

[10] Burke JF, Feng C, Skolarus LE (2019). Divergent poststroke outcomes for black patients: Lower mortality, but greater disability. Neurology.

[11] Cruz-Flores S, Rabinstein A, Biller J (2011). Racial-ethnic disparities in stroke care: the American experience: a statement for healthcare professionals from the American Heart Association/American Stroke Association. Stroke.

[12] Ghanchi H, Takayanagi A, Savla P (2020). Effects of the COVID-19 pandemic on stroke patients. Cureus.

[13] Bravata DM, Wells CK, Gulanski B (2005). Racial disparities in stroke risk factors: the impact of socioeconomic status. Stroke.

[14] Howard VJ, McClure LA, Kleindorfer DO (2016). Neighborhood socioeconomic index and stroke incidence in a national cohort of blacks and whites. Neurology.

[15] Howard VJ, Madsen TE, Kleindorfer DO (2019). Sex and race differences in the association of incident ischemic stroke with risk factors. JAMA Neurol.

[16] Yao J, Ghosh K, Perraillon MC, Cutler DM, Fang MC (2019). Trends and racial differences in first hospitalization for stroke and 30-day mortality in the US Medicare population from 1988 to 2013. Med Care.

[17] Park J-H, Ovbiagele B (2016). Association of black race with recurrent stroke risk. J Neurol Sci.

[18] Garg S, Kim L, Whitaker M (2020). Hospitalization rates and characteristics of patients hospitalized with laboratory-confirmed coronavirus disease 2019. MMWR Morb Mortal Wkly Rep.

[19] (2020). Nutrition and Health Are Closely Related - 2015-2020 Dietary Guidelines. https://health.gov/our-work/food-nutrition/2015-2020-dietary-guidelines/guidelines/introduction/nutrition-and-health-are-closely-related/.

[20] August KJ, Sorkin DH (2011). Racial/ethnic disparities in exercise and dietary behaviors of middle-aged and older adults. J Gen Intern Med.

[21] Zimmer MC, Rubio V, Kintziger KW, Barroso C (2019). Racial/ethnic disparities in dietary intake of U.S. children participating in WIC. Nutrients.

[22] Xu F, Cohen SA, Greaney ML, Hatfield DL, Greene GW (2019). Racial/ethnic disparities in US adolescents’ dietary quality and its modification by weight-related factors and physical activity. Int J Environ Res Public Health.

[23] Neuhouser ML, Thompson B, Coronado GD, Solomon CC (2004). Higher fat intake and lower fruit and vegetables intakes are associated with greater acculturation among Mexicans living in Washington State. J Am Diet Assoc.

[24] Avula A, Nalleballe K, Narula N (2020). COVID-19 presenting as stroke. Brain Behav Immun.

[25] Boehme AK, Luna J, Kulick ER, Kamel H, Elkind MSV (2018). Influenza-like illness as a trigger for ischemic stroke. Ann Clin Transl Neurol.

[26] Valderrama EV, Humbert K, Lord A, Frontera J, Yaghi S (2020). Severe acute respiratory syndrome coronavirus 2 infection and ischemic stroke. Stroke.

[27] Oudit GY, Kassiri Z, Jiang C (2009). SARS-coronavirus modulation of myocardial ACE2 expression and inflammation in patients with SARS. Eur J Clin Invest.

[28] Akhmerov A, Marbán E (2020). COVID-19 and the heart. Circ Res.

[29] Mao L, Jin H, Wang M (2020). Neurologic manifestations of hospitalized patients with coronavirus disease 2019 in Wuhan, China. JAMA Neurol.

[30] Fan H, Tang X, Song Y, Liu P, Chen Y (2020). Influence of COVID-19 on cerebrovascular disease and its possible mechanism. Neuropsychiatr Dis Treat.

